The article "Apolipoprotein E-Mimetic Peptide COG1410 Promotes Autophagy by Phosphorylating GSK-3β in Early Brain Injury Following Experimental Subarachnoid Hemorrhage" was retracted in 2025. Reasons: original data or images not available; unreliable results or conclusions; concerns about the data.

# Apolipoprotein E-Mimetic Peptide COG1410 Promotes Autophagy by Phosphorylating GSK-3β in Early Brain Injury Following Experimental Subarachnoid Hemorrhage

**DOI:** 10.3389/fnins.2018.00127

**Published:** 2018-03-05

**Authors:** Xinshen Li, Jianhua Peng, Jinwei Pang, Yue Wu, Xueping Huang, Yong Li, Jian Zhou, Long Gu, Xiaochuan Sun, Ligang Chen, Michael P. Vitek, Yong Jiang

**Affiliations:** ^1^Department of Neurosurgery, The Affiliated Hospital of Southwest Medical University, Luzhou, China; ^2^Department of Neurosurgery, The First Affiliated Hospital of Chongqing Medical University, Chongqing, China; ^3^Department of Neurosurgery, Luzhou People's Hospital, Luzhou, China; ^4^Medicine, Duke University Medical Center, Durham, NC, United States

**Keywords:** subarachnoid hemorrhage, early brain injury, autophagy, apolipoprotein E, glycogen synthase kinase 3 beta

## Abstract

COG1410, a mimetic peptide derived from the apolipoprotein E (apoE) receptor binding region, exerts positive effect on neurological deficits in early brain injury (EBI) after experimental subarachnoid hemorrhage (SAH). Currently the neuroprotective effect of COG1410 includes inhibiting BBB disruption, reducing neuronal apoptosis, and neuroinflammation. However, the effect and mechanism of COG1410 to subcellular organelles disorder have not been fully investigated. As the main pathway for recycling long-lived proteins and damaged organelles, neuronal autophagy is activated in SAH and exhibits neuroprotective effects by reducing the insults of EBI. Pharmacologically elevated autophagy usually contributes to alleviated brain injury, while few of the agents achieved clinical transformation. In this study, we explored the activation of autophagy during EBI by measuring the Beclin-1 and LC3B-II protein levels. Administration of COG1410 notably elevated the autophagic markers expression in neurons, simultaneously reversed the neurological deficits. Furthermore, the up-regulated autophagy by COG1410 was further promoted by p-GSK-3β agonist, whereas decreased by p-GSK-3β inhibitor. Taken together, these data suggest that the COG1410 might be a promising therapeutic strategy for EBI via promoting autophagy in SAH.

## Introduction

Subarachnoid hemorrhage (SAH) constitutes ~5% of all strokes with high mortality and morbidity (van Gijn and Rinkel, 2001; Bederson et al., 2009). The pathophysiological mechanism of SAH is not fully understood and recent studies mainly focus on early brain injury (EBI). EBI describes the brain injury typified by brain edema, elevated intracranial hypertension (ICP), and microcirculation compromise, within the first 72 h after SAH, which offers new approaches for the treatment of SAH (Kusaka et al., 2004).

The article "Apolipoprotein E-Mimetic Peptide COG1410 Promotes Autophagy by Phosphorylating GSK-3β in Early Brain Injury Following Experimental Subarachnoid Hemorrhage" was retracted in 2025. Reasons: original data or images not available; unreliable results or conclusions; concerns about the data.

During EBI, subcellular organelle functions become disordered, and the autophagy-lysosomal system is activated (Chen et al., 2015). As the main intracellular recycling system during conditions of starvation and various stressors, autophagy is a critical for neuronal survival (Mizushima and Komatsu, 2011). It is well-documented that a properly enhanced autophagy serves as neuroprotection, and mainly achieved through anti-inflammatory processes in acute brain injury (Galluzzi et al., 2016), pharmacologic upregulation of autophagy could slow the progression of Huntington disease and tauopathy models (Mizushima and Komatsu, 2011). Furthermore, several pharmacological activators of autophagy could effectively decrease acute brain injury in the SAH model (Galluzzi et al., 2016). However, few of those agents are feasible for clinical application.

The regulation of autophagy is a very complex process. As the direct downstream target of Akt, p-GSK-3β strongly induces the cytoplasmic autophagy (Park et al., 2013), and closely correlates with the alleviation of acute brain injury in SAH (Endo et al., 2006). Previous studies have shown that p-GSK-3β can be up-regulated by exogenous administration of apoE, thereby promoting neuronal survival (Han, 2004; Hayashi et al., 2007). However, apoE holoprotein is greatly restricted due to a molecular weight of 34 kDa, which makes it hard to cross the blood-brain barrier (BBB), thereby limiting its translational study.

Recently, a modified apolipoprotein E (apoE) mimetic peptide called COG1410 has been widely investigated. COG1410 is an apoE-mimetic peptide derived from the receptor-binding region, which could activate downstream receptors and produce beneficial effects. With a composition of apoE residues 138–149, and the modification of two amino residues, COG1410 could effectively cross the blood brain barrier (BBB), and potentially have a long duration for the treatment of SAH (Wu Y. et al., 2016). We recently showed that COG1410 could exert neuroprotective effects in EBI after experimental SAH, and activate downstream effectors including Akt (Pang et al., 2016; Wu Y. et al., 2016). Based on these observations, we aimed to investigate the effect of COG1410 on autophagy and the potential mechanism, during EBI after experimental SAH.

## Materials and methods

### Animals

A total of 130 adult male C57BL/6J mice were obtained from the Laboratory Animal Center of Chongqing Medical University, in which 98 mice were included in the experiment, and the other 32 mice died unexpectedly, as shown in the Supplementary Table 1. All the mice were aged 6–8 weeks, with a mean (±*SD*) weight of 20 ± 2 g. We followed the Guide for the Care and Use of Laboratory Animals of China, the number of mice was minimized as shown in the figures, and all the experimental mice were euthanized under deep anesthesia.

The article "Apolipoprotein E-Mimetic Peptide COG1410 Promotes Autophagy by Phosphorylating GSK-3β in Early Brain Injury Following Experimental Subarachnoid Hemorrhage" was retracted in 2025. Reasons: original data or images not available; unreliable results or conclusions; concerns about the data.

### Induction of SAH

To better mimic EBI process, we chose the endovascular perforation SAH model, as previously described (Peng et al., 2017). Briefly, mice were anesthetized with sodium pentobarbital and placed in a supine position. In the condition of mechanical ventilation, the right carotid artery was exposed, and a 5-0 filament was inserted into the isolated right external carotid artery to rupture the bifurcation of the right internal carotid artery (ICA). For the sham-operated mice, the filament entered the ICA but did not pierce the bifurcation. A sharp increase in ICP was a reliable parameter to detect the induction of SAH in the mouse model, and we mainly judged the success of SAH by monitoring the occurrence of the typical Cushing response.

### Animal groups

To evaluate the time course of autophagy in EBI, typical SAH models were induced, and after 6, 24, 48, and 72 h, the brain specimens were removed under deep anesthesia and randomly divided into five groups; the sham group was included, and each group comprised 5 mice based on the sample size calculation method (Charan and Kantharia, 2013). To observe the effect of the apoE-mimetic peptide, 53 mice were assigned to four groups: sham-operated, SAH operated for 24 h, saline-treated and COG1410-treated. In each group, 6 mice were used for western blotting measurement, 6 mice were used for immunofluorescence staining analysis, and the other mice was used for transmission electron microscope. For the mice in the COG1410 group, the peptide was injected via the tail vein immediately after SAH (2 mg/kg; Laskowitz et al., 2012). To explore the role of p-GSK-3β, 50 mice were divided into five groups: SAH+saline, SAH+COG1410, SAH+COG1410+DMSO, SAH+COG1410+OA, and SAH+COG1410+LY. In each group, 5 mice were used for western blotting measurement, and the other 5 mice were used for immunofluorescence staining analysis. In the last three groups, dimethyl sulfoxide (DMSO), okadaic acid (OA), and LY294002 (LY) were injected through the lateral ventricle, the injections were performed 15 min before the SAH operation, with a microsyringe fixed to the stereotaxic frame, the coordinates were −0.9 mm anteroposterior, ±1.5 mm mediolateral, and −3.5 mm dorsoventral from the bregma (Yang et al., 2014; Baker and Götz, 2016). We acquired the DMSO (sc-358801), OA (sc-3513A), and LY294002 (CAS 936487-67-1) from Santa Cruz Biotechnology.

### Measurements of neurological deficit and SAH severity

Garcia score (Garcia et al., 1995) consisted of six programs, the scores of the first three programs were 0–3, and the scores of the last three programs were 1–3. Each score was an integer, with the minimum score equal to 3 and the maximum score equal to 18.

The article "Apolipoprotein E-Mimetic Peptide COG1410 Promotes Autophagy by Phosphorylating GSK-3β in Early Brain Injury Following Experimental Subarachnoid Hemorrhage" was retracted in 2025. Reasons: original data or images not available; unreliable results or conclusions; concerns about the data.

A new grading system was utilized to grade the SAH model (Sugawara et al., 2008). Basal cisterns were divided into six segments, and each segment was graded from 0 to 3; grades 0, 1, 2, and 3 indicate no obvious subarachnoid blood clot, a minor blood clot, a moderate blood clot, and a large subarachnoid blood clot with an invisible cerebral arterial circle, respectively. Additionally, total grades of 0–7, 8–12, and 13–18 indicated mild, moderate, and severe SAH, respectively.

### Western blot

According to the previous reports, autophagy is more pronounced in the injured hemisphere, especially in the fronto-basal cortex (Lee et al., 2009), so the right hemisphere was quickly removed from the deeply anesthetized mouse and cut into pieces on ice. The pieces were subsequently homogenized in RIPA buffer that was previously mixed with a protease inhibitor (PMSF, 0.1 mM) and phosphatase inhibitor (sodium orthovanadate, 1 mM), and the mixture was centrifuged to obtain supernatant extracts. After the extracts were diluted with loading buffer, the protein extracts were transferred to polyvinylidene difluoride membranes after SDS-polyacrylamide gel electrophoresis and incubated with primary antibodies, which included Beclin-1 (1:500, Proteintech, 11306-1-AP), LC3B-II (1:200, Bioss Antibody, bs-4843R), p-GSK-3β (Serine 9) (1:200, Santa Cruz Biotechnology, sc-11757-R). Horseradish peroxidase-conjugated secondary antibodies were incubated with the primary antibodies, and the signal was detected by an ECL reagent (Thermo Scientific, #15168) and quantified using Image Lab software (Bio-Rad, ChemiDoc XRS+).

### Immunofluorescence staining

The brains were prefixed with 4% paraformaldehyde, dehydrated in the gradient concentration of sucrose solutions (20, 30%), and cut into frozen sections at the thickness of 6 μm. Then primary antibodies including Beclin-1 and LC3B-II, as well neuronal marker anti-NeuN (1:500, Merck Millipore, MAB377), were incubated on the sections. After the primary antibodies were labeled with fluorophore-conjugated secondary antibody, including anti-rabbit secondary antibody (1:200, Abbkine, Dylight 488) and anti-mouse secondary antibody (1:200, Abbkine, Dylight 549), the cell nuclei were counterstained with DAPI. The region of interest was observed with a fluorescence microscope (Nikon, C-HGFI), and the co-staining positive neurons were counted (MediaCybernetics, Image-ProPlus 6.0).

### Transmission electron microscopy

Mice were deeply anesthetized and sacrificed. Samples from the glutaraldehyde prefixed right fronto-basal cortex were then quickly acquired, cut into small samples, placed in 2.5% phosphate-buffered glutaraldehyde and stored overnight at 4°C. After dehydration in a graded ethanol series and subsequent fixation with osmium tetroxide, the samples were impregnated with epoxy resin and placed in an embedding medium. Sections that were 60-nm thick were sliced and stained with a saturated uranyl acetate solution, and the ultrastructure of neurons was observed using an electron microscope (JEOL, JEM-1400).

The article "Apolipoprotein E-Mimetic Peptide COG1410 Promotes Autophagy by Phosphorylating GSK-3β in Early Brain Injury Following Experimental Subarachnoid Hemorrhage" was retracted in 2025. Reasons: original data or images not available; unreliable results or conclusions; concerns about the data.

### Statistics

The statistics were analyzed by SPSS software 17.0 (SPSS Inc., Chicago, IL, USA), significance was assessed by one-way analysis of variance (ANOVA) followed by the LSD, and the data are presented as mean ± *SD*.

## Results

### Autophagy is activated and peaked at 24 H after experimental SAH

To investigate the alteration of autophagy (Figure 1A) in EBI after Experimental SAH, we measured a time course of Beclin-1 and LC3B-II, two commonly used autophagic markers (Liang et al., 2008; Mizushima and Yoshimori, 2014). According to protein quantification results, both the Beclin-1 and LC3B-II (Figure 1B) levels were elevated at 6 h and peaked at 24 h compared with the sham group. The results indicate that the autophagy level is enriched at 24-h, and thus, the time point is appropriate for the subsequent intervention study.

**Figure 1:** The time courses of autophagy in EBI after experimental SAH. **(A)** The relative densities of Beclin-1 and LC3B-II were quantified by western blot. **(B)** The band intensities were increased in the SAH-6H group and peaked in the SAH-24H group, as the quantitative results shown. ^*^P < 0.05 and ^##^*P* < 0.01 vs. sham group, *n* = 5 animals per group.

### The specimen, SAH grade, and neurological score of SAH models

In Figure 2A, blood clots were evident in the ventral subarachnoid space of SAH mice, but not in the control animals. The boxed region represents the right fronto-basal cortex areas for immunofluorescence staining and transmission electron microscopy. In Figure 2B, the SAH grade of mice in SAH group, SAH+Saline group, and SAH+COG1410 group were higher than that in Sham group, but were not statistically different when they compared with each other. In Figure 2C, neurological scores of the SAH group were strongly decreased relative to the sham group, but the neurological dysfunction can be significantly attenuated by the administration of COG1410. These data suggest that the SAH models are typical and steady, and the neurologic defect of mice models could be improved by COG1410 treatment.

The article "Apolipoprotein E-Mimetic Peptide COG1410 Promotes Autophagy by Phosphorylating GSK-3β in Early Brain Injury Following Experimental Subarachnoid Hemorrhage" was retracted in 2025. Reasons: original data or images not available; unreliable results or conclusions; concerns about the data.

**Figure 2:** The Specimen, SAH Grade, and Neurological Score of SAH Models. **(A)** For the sham-operated mice, there were no distributions of hemorrhage or blood clot in the basal pool (The left picture), but for the typical SAH models, the blood clots distributed into the basal cistern and nearly covered the circle of Willis, as indicated by black arrow heads (The right picture). The boxed region represents the right fronto-basal cortex area, which is the region of interest for immunofluorescence microscopy and transmission electron microscopy. **(B)** The total SAH grade in the SAH, SAH+saline and SAH+COG1410 groups showed no significant difference, the grades were 15.33 ± 1.21, 14.33 ± 1.63, and 13.83 ± 1.83, respectively (*n* = 6 animals per group). **(C)** Mice subjected to SAH for 24 h had significantly low Garcia scores compared with the sham-operated mice (SAH: 11.20 ± 2.05, vs. sham: 16.40 ± 1.14); after administration of COG1410, the neurological score significantly increased to 15.20 ± 0.84 (*n* = 6 animals per group). ^**^P < 0.01 vs. sham group; ^##^*P* < 0.01 vs. SAH group.

### Transmission electron microscopy of COG1410 promoted neuron autophagy

Through analysis of electron microscope images captured by a blinded observer, we found that subcellular structures, including the nuclear membrane, mitochondria and endoplasmic reticulum, were relatively intact in the sham group (Figure 3A). After experimental SAH, the mitochondria began to swell in the neurons, the nuclear membrane became shrunken, and the early autolysosome was evident (Figure 3B). In the saline group, the multiple-membrane autophagosome became evident and contained cytoplasmic disintegration (Figure 3C). After administration of COG1410, autophagy was increased, and neurons showed both autophagosomes and autolysosomes in the cytoplasm (Figure 3D). These results suggest that the administration of COG1410 could enhance neuronal autophagy, which may contribute to the breakdown of injured cellular components after SAH.

**Figure 3:** The subcellular structure and autophagic activity in neurons. **(A)** The complete nuclear membrane (white arrow head), healthy endoplasmic reticulum (white pentagram) and mitochondria (white arrows) in the relatively normal neuron of the sham group. **(B)** In the neuron of the SAH model, the nuclear membrane was shrunken, mitochondria were typically swollen and deformed (open white arrow), and the early autolysosome began to form (white asterisk). **(C)** In SAH+saline group, the multiple-membrane autophagosome (black arrows) appeared in the neuronal cytoplasm. **(D)** In the SAH+COG1410 group, both the typical autophagosomes (black arrows) and autolysosome (white asterisk) were visible in the neuron.

The article "Apolipoprotein E-Mimetic Peptide COG1410 Promotes Autophagy by Phosphorylating GSK-3β in Early Brain Injury Following Experimental Subarachnoid Hemorrhage" was retracted in 2025. Reasons: original data or images not available; unreliable results or conclusions; concerns about the data.

### COG1410 improves autophagy level

Beclin-1 and LC3B-II levels in right brain hemispheres, as quantified by western blot, were prominently elevated after SAH, and then picked up at 24 h. COG1410 treatment significantly increased Beclin-1 and LC3B-II levels when compared with the saline-treated group 24 h after SAH (Figures 4A,B). To confirm the major cell type of Beclin-1 and LC3B-II, immunofluorescence analysis that involved double staining with NeuN was performed, and the results were consistent with the quantitative data from the western blot analysis (Figures 4C–E). These data indicate that the administration of COG1410 elevates autophagy in the injured brain and in neuronal cells of an SAH model.

**Figure 4:** Autophagy of mice brain and neuron with the administration of COG1410. **(A,B)** The band intensities of Beclin-1 and LC3B-II were conspicuously increased in the SAH group compared with the Sham group, and further enhanced in the COG1410 group compared to the SAH group. No significant differences were observed between the SAH+Saline group and the SAH group, the relevant results are shown in the quantification (*n* = 6 animals per group). **(C–E)** The co-staining of NeuN with Beclin-1 and LC3B-II is indicated by white arrow heads and amplified in the upper-right corners of the merged images, and the relevant bio-markers are shown in the two smaller pictures below. The number of co-stained cells was also prominently increased in the SAH group and increased further in the SAH+COG1410 group (*n* = 6 animals per group). ^**^P < 0.01 vs. the sham group; ^#^*P* < 0.05 vs. the SAH group.

### The ApoE-mimetic peptide elevates p-GSK-3β level

Given that the phosphorylation of GSK-3β is an important regulator for autophagy (Zhou et al., 2011; Park et al., 2013), we conducted western blot (Figure 5A) and immunofluorescence (Figure 5D) analyses for p-GSK-3β in the right cerebral hemisphere. According to the quantification results (Figure 5B), the total p-GSK-3β level increased sharply in the SAH group and administration of COG1410 further increased the p-GSK-3β level of ipsilateral hemisphere compared with SAH+Saline group. The number of co-staining neurons was also augmented in the SAH group and further increased by the administration of COG1410 (Figure 5C). This shows that p-GSK-3β expression in the brain and neurons is also elevated after treatment with COG1410, which is closely related to the altered autophagy by administration of COG1410.

**Figure 5:** p-GSK-3β level of mice brain and neuron after administrating COG1410. **(A,B)** In the western blot analysis, p-GSK-3β level was increased substantially in the SAH group compared to the Sham group, and enhanced further in the SAH+COG1410 group compared to the SAH+Saline group, while there were no major differences between the SAH+Saline group and SAH group (*n* = 6 animals per group). **(C,D)** The co-staining of NeuN and p-GSK-3β indicates that the expression of p-GSK-3β was further elevated by COG1410, as the analysis result shown (*n* = 6 animals per group). ^**^P < 0.01 vs. the sham group; ^#^*P* < 0.05 vs. the SAH group.

The article "Apolipoprotein E-Mimetic Peptide COG1410 Promotes Autophagy by Phosphorylating GSK-3β in Early Brain Injury Following Experimental Subarachnoid Hemorrhage" was retracted in 2025. Reasons: original data or images not available; unreliable results or conclusions; concerns about the data.

### The phosphorylation and dephosphorylation of GSK-3β were effectively achieved

As the main inactive state of GSK-3β, p-GSK-3β could be effectively achieved by a serine inhibitor OA, and greatly depressed by the PI3K inhibitor LY (Park et al., 2013). In western blot, the p-GSK-3β level was increased after administrating COG1410. Furthermore, the p-GSK-3β level was significantly elevated after the OA injection but apparently reduced after the LY injection (Figures 6A,B). Immunofluorescence further supported the results of western blot (Figures 6C,D).

**Figure 6:** The Phosphorylation and dephosphorylation of GSK-3β. **(A,B)** The band density of p-GSK-3β was noticeably increased in the SAH+COG1410 group compared to the SAH+Saline group. The OA injection increased the p-GSK-3β level sharply, whereas the level decreased linearly in LY-injected group compared with the DMSO injecting mice (*n* = 5 animals per group). **(C,D)** The positive double staining neurons were counted and quantified; the cell number increased noticeably in the SAH+COG1410 group. Furthermore, the co-staining-positive neurons increased drastically in the SAH+COG1410+OA group, but decreased noticeably in the SAH+COG1410+LY group (*n* = 5 animals per group). ^*^P < 0.05 vs. the SAH+saline group; ^##^*P* < 0.01 vs. the SAH+COG1410 group; ^&&^*P* < 0.01 vs. the SAH+COG1410 group.

### COG1410 promotes neuronal autophagy by promoting the phosphorylation of GSK-3β

COG1410 increased the protein levels of autophagy, and the band densities of Beclin-1 and LC3B-II were both further promoted in the SAH+COG1410+OA group. However, the protein level showed a striking decrease in the SAH+COG1410+LY group (Figures 7A,B). Additionally, the immunofluorescence staining for the co-staining analysis was also consistent with the western blot analysis (Figures 7C–E).

**Figure 7:** Effect of p-GSK-3β to the COG1410 promoted neuron autophagy. **(A,B)** Western blot analysis of Beclin-1 and LC3B-II indicates increased band densities for the SAH+COG1410 group compared to the SAH+Saline group, and the densities increased further in the SAH+COG1410+OA group but decreased dramatically in the SAH+COG1410+LY group compared with the SAH+COG1410+DMSO group, as the quantitative results shown (*n* = 5 animals per group). **(C–E)** The double staining of NeuN with Beclin-1 and LC3B-II yielded similar results as the analysis results shown (*n* = 5 animals per group). ^*^P < 0.05 vs. the SAH+saline group; ##*P* < 0.01 vs. the SAH+COG1410 group; &&*P* < 0.01 vs. the SAH+COG1410 group.

The article "Apolipoprotein E-Mimetic Peptide COG1410 Promotes Autophagy by Phosphorylating GSK-3β in Early Brain Injury Following Experimental Subarachnoid Hemorrhage" was retracted in 2025. Reasons: original data or images not available; unreliable results or conclusions; concerns about the data.

## Discussion

In this present study, we assessed the neuroprotective effects of COG1410 and explored the possible underlying mechanism of COG1410 in neuronal autophagy during EBI after SAH. With the administration of apoE-mimetic peptide COG1410, the autophagy was further promoted, accompanied by the improvement of neurological score. Additionally, we confirmed that the autophagy-promoting effect of COG1410 can be achieved by the phosphorylation of GSK-3β, both in the injured brain tissue and neuronal cell.

As an essential pathway to recycle long-lived proteins and damaged organelles (Levine and Klionsky, 2004; Wu H. et al., 2016), autophagy is ubiquitously present in various diseases, and the current studies consider brain autophagy as important for neuronal survival in SAH (Galluzzi et al., 2016). The pharmacological promotion of autophagy significantly alleviates the acute brain injury of SAH (Jing et al., 2012; Zhao et al., 2013; Chen et al., 2014; Shao et al., 2014), whereas inhibition of autophagy using either 3-MA or wortmannincan worsen the brain injury (Jing et al., 2012; Zhao et al., 2013) or eliminate the neuroprotective effects of enhanced autophagy (Shao et al., 2014). These observations suggest that properly augmented autophagy levels benefit neuronal survival and may affect the prognosis of EBI. In the current study, administration of COG1410 increased autophagic markers and p-GSK-3β levels, and the neurological scores of SAH models were improved. This may suggest that COG1410-promoted autophagy is a protective intervention for SAH models, and points to the potential involvement of p-GSK-3β in the process.

As the downstream effector kinase of Akt, p-GSK-3β could be increased by the phosphorylation of Akt (Wang et al., 2017), and promote the survival of damaged neurons (Hetman et al., 2000; Liang and Chuang, 2007; Collino et al., 2008). The Akt/GSK-3β signaling could also alleviate acute brain injury following experimental SAH (Endo et al., 2006). Our previous study demonstrated that COG1410 could effectively promote the phosphorylation of Akt (Wu Y. et al., 2016). Furthermore, phosphorylated GSK-3β profoundly induces the occurrence of neuronal autophagy (Zhou et al., 2011). Thus, we hypothesized that COG1410 promotes autophagy by indirectly facilitating the phosphorylation of GSK-3β. In this study, the apoE analog could promote autophagy when GSK-3β was phosphorylated by OA, but depress autophagy when GSK-3β was dephosphorylated by LY. In fact, the exogenous administrated apoE effectively phosphorylates GSK-3β through LRP1/GSK-3β pathway, and significantly activates downstream pathways by binding to LRP-1 [8, 34]. Therefore, COG1410 may also promote the phosphorylation of GSK-3β through LRP1/GSK-3β pathway, but it remains further confirmation.

The article "Apolipoprotein E-Mimetic Peptide COG1410 Promotes Autophagy by Phosphorylating GSK-3β in Early Brain Injury Following Experimental Subarachnoid Hemorrhage" was retracted in 2025. Reasons: original data or images not available; unreliable results or conclusions; concerns about the data.

According to our previous study, among the three subtypes of apoE protein-coding gene (APOE), the APOE4 isoform is unfavorable for neuronal survival compared to the APOE3 isoform (Jiang et al., 2007, 2015), while COG1410 is derived from the apoE-receptor-binding region and free from the APOE polymorphism. Additionally, COG1410 can effectively pass through the BBB. By reducing the number of activated microglia, COG1410 effectively alleviates the neuroinflammatory response in TBI (Jiang and Brody, 2012), and decreases the neurologic deficit during intracranial hemorrhage (Laskowitz et al., 2012). As a neuroprotective agent, COG1410 can inhibit BBB disruption with the activating of CypA/NF-κB/MMP-9 pathway, and reduce apoptosis and neuroinflammation by activating downstream effectors in EBI following SAH (Pang et al., 2016; Wu Y. et al., 2016). From these facts, COG1410 retains the receptor-binding property of apoE holoprotein, the peptides could activate the downstream effectors, and produce neuroprotection in EBI after experimental SAH.

Although these data indicate the potential neuroprotection and the possible mechanism of COG1410-promoted autophagy, our study has some limitations. The other GSK isoforms are incompletely detected by the experiments, and the neurological effect of COG1410 in the late phase of SAH is worthy of future studies. Additionally, further investigation needs to be performed in the safety, efficacy, and clinical study of the apoE-mimetic peptide.

## Author contributions

XL, YJ: Designed the study; XL, JHP, JWP, XH, YL, JZ, LG: Contributed to the sample preparation, data collection, and data analysis; YW, XS, LC, YJ: Directed the experiments; COG1410 was a gift from MV; XL, JHP, JWP: Wrote the manuscript together, and all the authors reviewed the manuscript.

### Conflict of interest statement

The authors declare that the research was conducted in the absence of any commercial or financial relationships that could be construed as a potential conflict of interest.

## Supplementary material

Supplementary Table 1 **Experimental design and mortality rate**.
